# Effects of microRNA-374 on proliferation, migration, invasion, and apoptosis of human SCC cells by targeting Gadd45a through P53 signaling pathway

**DOI:** 10.1042/BSR20170710

**Published:** 2017-08-04

**Authors:** Xiao-Jing Li, Zhi-Feng Li, Jiu-Jiang Wang, Zhao Han, Zhao Liu, Bao-Guo Liu

**Affiliations:** Department of Dermatology, Affiliated Hospital of Hebei Engineering University, Handan 056002, P.R. China

**Keywords:** Apoptosis, Gadd45a, MicroRNA-374, P53 signaling pathway, Proliferation, Squamous carcinoma cells

## Abstract

The present study investigated the effects of microRNA-374 (miR-374) on human squamous cell carcinoma (SCC) cell proliferation, migration, invasion, and apoptosis through P53 signaling pathway by targeting growth arrest and DNA-damage-inducible protein 45 α (Gadd45a). Skin samples were collected from patients with skin SCC and normal skin samples. Expression of miR-374, Gadd45a, P53, P73, P16, c-myc, bcl-2, Bax, caspase-3, and caspase-9 were detected using quantitative real-time polymerase chain reaction (qRT-PCR) and Western blotting. A431 and SCL-1 cells were divided into blank, negative control (NC), miR-374 mimics, miR374 inhibitors, siRNA–Gadd45a, and miR-374 inhibitors + siRNA–Gadd45a groups. Their proliferation, migration, invasion, cell cycle, and apoptosis were evaluated by 3-[4,5-dimethylthiazol-2-yl]-2,5 diphenyl tetrazolium bromide (MTT) assay, scratch test, Transwell assay, and flow cytometry. SCC skin tissues exhibited decreased expression of miR-374, P73, P16, Bax caspase-3 and caspase-9, and increased levels of Gadd45a, P53, c-myc, and Bcl-2 compared with the normal skin tissues. The miR-374 inhibitors group exhibited decreased expression of miR-374, P73, P16, Bax caspase-3 and caspase-9, and increased expression of Gadd45a, P53, c-myc, and Bcl-2, enhanced cell proliferation, migration, and invasion, and reduced apoptosis compared with the blank and NC groups; the miR-374 mimics group followed opposite trends. Compared with the blank and NC groups, the miR-374 inhibitors + siRNA–Gadd45a group showed decreased miR-374 level; the siRNA–Gadd45a group showed elevated levels of P73, P16, Bax, caspase-3 and caspase-9, decreased levels of Gadd45a, P53, c-myc, and Bcl-2, reduced cell proliferation, migration, and invasion, and accelerated apoptosis. miR-374 induces apoptosis and inhibits proliferation, migration, and invasion of SCC cells through P53 signaling pathway by down-regulating Gadd45a.

## Introduction

Squamous cell carcinoma (SCC) is a type of epithelial cancer with relatively high morbidity, ranked as the second most common type among non-melanoma skin cancers [1]. The strongest risk factor of SCC is exposure to ultraviolet (UV) light, and the most common disease occurrence sites are the sun-exposed neck and head [2]. Biological behavior of SCC is usually related to pathological factors like histological grade, size, vascular and perineural invasion, and depth of infiltration [3]. It is trivial to understand the transformation mechanisms of both cell types in order to find novel ways for permanent prevention and treatment of SCC [4]. It has been proved that growth arrest and DNA-damage-inducible protein 45 α (Gadd45a) can protect against UV irradiation-induced skin tumors, and promote stress signaling and apoptosis via mitogen-activated protein kinase (MAPK) and P53 pathways [5]. Moreover, it has suggested that Gadd45a plays a significant role in the metastasis of oral SCC (OSCC) by regulating the bioactivity of those tumor cells [6]. Therefore, Gadd45a might be a new biomarker for the prediction of clinical outcome of SCC.

Gadd45a is the first well-defined downstream gene of P53, and is regulated by P53 tumor suppressor, which can be triggered by all kinds of DNA-damaging agents and plays a key role in the control of DNA repair process, signaling transduction, and cell cycle checkpoint [7]. It has also revealed that Gadd45a is critical in the demethylation of gene-specific active DNA during the differentiation of adult stem cells [8]. P53, the ‘guardian of the genome’, is involved in many reaction mechanisms acting as an advanced sentinel for DNA impairment, and other cell stresses, including starvation, oncogene activation, hypoxia, altered ribosomal and mitochondrial biogenesis, denuded telomeres, or spindle poisons [9]. During the event of DNA damage, P53 is capable of either promoting cell survival by activating cell cycle arrest or senescence and DNA repair to maintain genomic integrity or conducting cell apoptosis in order to eliminate extensively damaged cells, both of which are executed depending on different signaling pathways of P53 downstream [10]. A previous study found that expression profiling of skin SCC with perineural invasion implicated the P53 pathway and its functioning [2]. microRNAs (miRs) are vital regulators of many pathological and physiological processes, including metastasis and tumorigenesis [11]. In addition, miR-374 has been suggested to be a novel biomarker for determining the most appropriate treatment for cancer and a novel radiation sensitizer for carbon ion beam radiotherapy [12]. In the present study, we aim to investigate the effects of miR-374 on proliferation, migration, invasion, and apoptosis of human SCC cells by targeting Gadd45a through the P53 signaling pathway.

## Materials and methods

### Ethic statement

Signed informed consents were obtained from all patients participating in the study. The experiment was approved by the Clinical Ethics Committee of the Affiliated Hospital of Hebei Engineering University.

### Study subjects

A total of 265 skin SCC samples (SCC group) were selected from patients undergoing clinical physical health checks at the Affiliated Hospital of Hebei Engineering University from 2006 to 2015. The study included 155 males and 110 females, with a calculated mean age of 65.47 ± 12.85 years (age of patients ranged from 40 to 82 years). A total of 103 cases in the SCC group had detailed medical history, and all of them were originated single. The observed tumor diameter ranged from 1 to 10 cm, and area of the largest lesion was approximately 10 cm × 10 cm. Among them, the skin lesions had a diameter smaller than 1 cm in 78 cases, 1–4.9 cm in 103 cases, and 5–10 cm in 84 cases. SCC skin was secondary to chronic ulcer in 71 cases, scars in 60 cases, subcutaneous mass in 38 cases (caused by repeated physical stimulation), lichen planus in 31 cases, chronic skin inflammation in 45 cases, and unknown causes in 20 cases. A microscope was used to observe pathological changes in the lesions, and observations revealed that proliferated cell epithelium penetrated the basement membrane and formed cancer nests in the shape of irregular elongated strip. In accordance with the differentiation degree [13], there were 125 high differentiation cases, 78 middle differentiation cases, and 62 low differentiation cases. A total of 102 normal skin samples (normal group) were selected from 57 males and 45 females, with a calculated mean age of 58.07 ± 10.01 years (age of patients ranged from 15 to 65 years). Skin samples were obtained from the head, face, limbs, and the trunk of the patients. The participants did not undergo radiotherapy, chemotherapy, physical therapy, or other special treatments before the operation and had no history of immunological or systemic diseases. All SCC and normal tissue samples were sliced into small pieces and preserved in frozen pipes with liquid nitrogen, and refrigerated in an ice box at −80°C.

### Hematoxylin–eosin staining

All tissue samples were fixed with formaldehyde, embedded with paraffin, cut into 4-μm-thick slices, and stained with hematoxylin–eosin (HE). Next, the slices were dewaxed using xylene two times (15 min each) and washed with absolute alcohol two times (5 min each). Subsequently, the slices were rinsed with 90% alcohol for 5 min and 80% alcohol for 5 min, and washed with water for 5 min. Hematoxylin staining was conducted for 5 min and the slices were washed with running water till blue coloration was observed. Next, color separation with 1% hydrochloric (HCl)–ethanol, washing with water till blue coloration, dehydration and clearing and mounting with 80% alcohol for 5 min, 90% alcohol for 5 min, absolute alcohol two times (5 min each), xylene two times (15 min each), and mounting with resin were performed orderly. Subsequently, the slices were observed under a microscope and photographed, and morphologically analyzed at ×200 magnification. The experiment was repeated three times.

### Immunohistochemistry

Approximately 10% formalin-fixed samples were paraffin-embedded and cut up into 4-μm-thick slices. The slices were placed into a 60°C incubator for 1 h, conventionally dewaxed with xylene, and dehydrated using gradient alcohol, followed by repair by citric acid in an autoclave. Next, the slices were heated at 1800 W until air injection, followed by heating at 1000 W for 2 min, natural cooling for 10 min, and washing with water for 10 min and subsequently the slices were gradually cooled with water after opening the lid of the autoclave. The slices were rinsed with 0.2 mol/l phosphate buffer solution (PBS) (pH 7.4) three times (5 min each), dried, and supplemented with polyclonal antibody (rabbit anti-human) Gadd45a (dilution ratio of 1:100, ab180768, Santa Cruz Biotechnology, Inc., Santa Cruz, CA, U.S.A.), and incubated at 4°C overnight, rinsed with 0.2 mol/l PBS (pH 7.4) three times (5 min each) and dried. Next, secondary antibodies labeled with peroxidase were supplemented into the slices, followed by incubation at room temperature for 15 min. In order to prepare the developer, one drop each of A, B, and C reagents of diaminobenzidine (DAB) solution (DA1010, Beijing Solarbio Science & Technology Co., Ltd., Beijing, China) was added and mixed well in 1 ml of distilled water, and preserved in the refrigerator at 4°C. The slices were rinsed again in 0.2 mol/l PBS (pH 7.4) three times (5 min each), and after DAB development, the slices were set aside at room temperature for 8 min devoid of light. The slices were visualized using a light microscope after washing with water, dyeing with hematoxylin, dehydration, clearing, and mounting. Cells identified by blue or light blue coloration in the nucleus were regarded as negative cells, and yellow or brown colored cells were regarded as positive cells. Three non-overlapping visual fields (×200) with equal areas were randomly chosen for each slice, and Nikon image analysis software (Nikon Vision Co. Ltd., Tokyo, Japan) was used in order to count the number of positive cells. The computational formula was as follows: percentage of positive cells = (number of positive cells/total cell number) × 100%.

### Quantitative real-time polymerase chain reaction

Total RNA in the tissue specimens was extracted using a RNA extraction kit (Art. No.: 10296010, Invitrogen Company, Shanghai, China). After detection of RNA purity and integrity, a PrimeScript RT kit (RR014A, TaKaRa Bio Inc., Beijing, China) was used to reverse transcribe the RNA into cDNA using a 10 μl reverse transcription (RT) system and the reaction conditions were as follows: 37°C, 15 min (three times, RT reaction), 85°C for 5 s (inactivation of reverse transcriptase). The primer sequences (miR-374, Gadd45a, P53, P73, P16, c-myc, Bcl-2, and Bax, internal reference U6, and glyceraldehyde-phosphate dehydrogenase (GAPDH)) were synthetized by the TaKaRa company (Table 1). The reaction system contents were as follows: 10 µl of SYBR Premix Ex Taq^TM^ II, 0.4 µl of PCR Forward Primer (10 µM), 0.4 µl of PCR Reverse Primer (10 µM), 2 µl of DNA template, and 7.2 µl of sterile purified water. Following the instructions of the PCR kit (KR011A1, TIANGEN Biotechnology Co. Ltd, Beijing, China), the reaction conditions were as follows: 5 min cycles at 95°C for pre-denaturation (30 cycles), 10 s at 95°C for denaturation, 57°C and 72°C in turn for annealing, then 10 min at 72°C for extension, and 5 min at 4°C for extension. The relative expression of miR-374 was calculated using U6 as the internal reference. In addition, GAPDH was used as the internal reference to calculate the relative expression of other mentioned genes including Gadd45a, P53, P73, P16, c-myc, Bcl-2, and Bax, which were compared using the 2^−△△*C*^t method according to the *C*_t_ value analyzed by LightCycler.

**Table 1:** Primer sequences for quantitative real-time polymerase chain reaction (qRT-PCR)

Gene	Primer sequences (5′-3′)
miR-374	Forward: UUAUAAUACAACCUGAUAAGUG
	Reverse: CUUAUCAGAUUGUAUUGUAAUU
Gadd45a	Forward: CCGAAAGGATGGATAAGGTGGG
	Reverse: CATGTAGCGACTTTCCCGGCAA
P53	Forward: ACATCTGGCCTTGAAACCAC
	Reverse: CGAGACCCAGTCTCAAAGAA
P73	Forward: TGGAACCAGACAGCACCTACTTCG
	Reverse: TGCTGGAAAGTGACCTCAAAGTGG
P16	Forward: TGGAGCCTTCGGCTGACT
	Reverse: CTATGCGGGCATGGTTACTG
c-myc	Forward: GCCACGTCTCCACACATCAG
	Reverse: TCTTGGCAGCAGGATAGTCCTT
Bcl-2	Forward: CGCCCTGTGGATGACTGAGTA
	Reverse: GGGCCGTACAGTTCCACAAAG
Bax	Forward: GGTTTCATCCAGGATCGAGACGG
	Reverse: ACAAAGATGGTCACGGTCTGCC
U6	Forward: GCTTCGGCAGCACATATACTAAAAT
	Reverse: CGCTTCACGAATTTGCGTGTCAT
GAPDH	Forward: CCAGCCGAGCCACATCGCTC
	Reverse: ATGAGCCCCAGCCTTCTCCAT

Abbreviation: miR-374, microRNA-374.

### Dual-luciferase reporter gene assay

The biological prediction website, www.microRNA.org, identified that Gadd45a was a direct target of miR-374. The synthetic Gadd45a 3′-UTR gene segment was introduced into pMIR-reporter (Promega, Madison, WI, U.S.A.) using restriction enzymes, SpeI and HindIII. The mutation site in complementary sequences of wild-type (WT) Gadd45a was designed. After restriction endonuclease digestion, the target segments were inserted into the pMIR-reporter plasmids using the T4 DNA ligase. The identified luciferase reporter plasmids WT and mutant-type (MUT) were respectively co-transfected into HEK-293T cells (Shanghai North Connaught Biotechnology Co. Ltd., Shanghai, China) with miR-374. After 48 h, the cells were collected and lysed, and luciferase activity was detected using a luciferase assay kit.

### Cell culture, transfection, and grouping

Human normal skin cells and SCC skin cell line A431 (CRL-1555, Biomics Technology Co., Ltd., Nantong, Jiangsu) and SCL-1 (JN-A2017, Shanghai Ji Ning Industrial Co., Ltd., Shanghai, China) were adherently cultured in Dulbecco’s minimum essential medium (DMEM) with high glucose containing 100 µg/ml penicillin, 10% fetal bovine serum (FBS), and 100 µg/ml streptomycin. All cells were kept in saturated humidity and 5% CO_2_ incubators at 37°C. The medium solution was changed every 1–2 days and the cells adhered to the base of the dish, forming a monolayer. Once the cells settled at the bottom, 0.25% trypsin digestion was used for cell digestion and the cells in logarithmic phase of growth were selected for further experimentation.

Third generation cells were selected and divided into normal, blank (with no transfection), negative control (NC), miR-374 mimics (transfected with miR-374 mimics), miR-374 inhibitors (transfected with miR-374 inhibitors), siRNA–Gadd45a (transfected with siRNA–Gadd45a), and miR-374 inhibitors + siRNA–Gadd45a groups (transfected with miR-374 inhibitors and siRNA–Gadd45a). The SCC skin cells in logarithmic phase of growth were inoculated in a six-well plate and allowed to reach 30–50% confluency, followed by transfection in accordance with the criteria of the lipofectamine 2000 transfection kit (Invitrogen Inc., Carlsbad, CA, U.S.A.). Each sequence in different groups and 5 µl of lipofectamine 2000 were respectively diluted using 250 µl of serum-free Opti-MEM medium (Gibco BRL, Grand Island, NY, U.S.A.), followed by mixing and incubation at room temperature for 5 min. The aforementioned two complexes were fully mixed, and incubated at room temperature for 20 min and subsequently added in culture plates. After that, the cells were placed in a 5% CO_2_ incubator at 37°C for 6–8 h and then cultured in complete medium for 24–48 h.

### Western blotting

After 48 h of cell transfection and grouping, human SCC cell line A431 and SCL-1 in each group were supplemented with radioimmunoprecipitation assay (RIPA) protein lysate (PS0013, TIANGEN Biotechnology Co. Ltd., Beijing, China), and lysed for 30 min, followed by centrifugation at a rate of 3000 rev/min for 20 min at 4°C. The obtained liquid supernatant was separated and sub-packed and preserved at −80°C after detection of the total protein content according to the bicinchoninic acid (BCA) Protein Assay Kit. Protein (50 µg) from each group was collected and supplemented with a protein denaturant (38249090, Sibas biotechnology company, Shanghai, China). Following, the protein was denatured for 10 min after boiling, separated using sodium dodecyl sulfate/polyacrylamide gel electrophoresis (SDS/PAGE), and then moved to nitrocellulose membranes from SDS/PAGE by electrophoretic transfer. The nitrocellulose membranes in each group were blocked in phosphate-buffered saline Tween-20 (PBST) containing 10% non-fat milk powder at 4°C overnight, rinsed in PBST three times (5 min each), and correspondingly added with primary antibodies of rabbit anti-human (Gadd45a: ab76664, dilution ratio 1:100; P53: ab26, dilution ratio 1:200; P73: ab40658, dilution ratio 1:200; P16: ab51243, dilution ratio 1:100; c-myc: ab30272, dilution ratio 1:10000; Bcl-2: ab32142, dilution ratio 1:300; Bax: ab32503, dilution ratio 1:200; caspase-3: ab2171, dilution ratio 1:500; and caspase-9: ab32539, dilution ratio 1:1000) (Abcam Inc. Cambridge, MA, U.S.A.) and subsequently incubated for 2 h at 37°C. Next, the membranes was washed in PBST three times (10 min each), and supplemented with goat anti-rabbit secondary antibodies immunoglobulin G (IgG) (dilution ratio 1:1000, DF109489, Yao Yun Biological Technology Co., Ltd., Shanghai, China) and incubated for 2 h at 37°C, and washed in PBST three times (10 min each). Chemiluminescence reagent (ECL kit, 36208ES60, Amersham Life Sciences Company, Arlington Heights, IL, U.S.A.) was adopted for development of slices, and the gray value analysis was performed using the ImageJ software. Using GAPDH as the internal reference, the ratio of gray value between the target band and internal reference band was regarded as the relative expression of the aforementioned proteins. Experiments for each sample were repeated three times.

### 3-[4,5-dimethylthiazol-2-yl]-2,5 diphenyl tetrazolium bromide assay

Cells in the logarithmic phase of growth and good growth-condition were seeded in a 96-well plate (1 × 10^4^ cells and 200 μl of medium in each well). A431 and SCL-1 cells adhered to walls of the well and were subsequently cultured in a 5% CO_2_ incubator at 37°C for 24, 48, and 72 h. Twenty microliters of 3-[4,5-dimethylthiazol-2-yl]-2,5 diphenyl tetrazolium bromide (MTT) solution (5 mg/ml) was added to each well, followed by incubation for 4 h at 37°C, and consequently, the supernatant was discarded. Next, 150 μl of dimethyl sulfoxide (DMSO) solution was added to each well, and the plates were vibrated for 10 min. The optical density (OD) value of each well was detected at a wavelength of 490 nm. The experiments were repeated three times and the mean value was recorded.

### Scratch test

Cells in the logarithmic phase of growth from each group were collected and seeded in a six-well plate (1 × 10^6^ cells per well) and placed in a 5% CO_2_ incubator at 37°C and allowed to reach 95% confluence. Micro pipette tips (20 μl) were used to make vertical scratches in the six-well plate. A D-hanks solution was used to remove the falling cells and the remaining cells were allowed to culture in a serum-free culture medium. At 0 and 36 h after scratching, three fields were selected in each group and photographed using a phase contrast microscope (×100) in order to compare the scratch-healing differences among groups, which represent cell migration and healing abilities.

### Transwell assay

Forty-eight hours following transfection, the cells were starved in a serum-free medium for 12 h, digested, and rinsed two times in PBS, then re-suspended in a serum-free medium Opti-MEMI containing 10 g/l bovine serum albumin (BSA) (31985-070, Invitrogen Inc., Carlsbad, CA, U.S.A.). The cell density was adjusted to 2 × 10^6^/ml, and the cells were inoculated in a 24-well plate 8-μm chamber (3413, Corning Inc, Corning, NY, U.S.A.), with three chambers in each group. Before the experiment, 50 μl of matrigel (40111ES08, Sigma–Aldrich Chemical Company, St Louis MO, U.S.A.) was added to each chamber. After 48 h, the apical chambers of Transwell chambers were dispensed with 200 μl of single cell suspension (4 × 10^4^ cells); meanwhile, 650 μl of G-DMEM containing 10% FBS was added to the basolateral chambers of Transwell chambers, and kept in a 5% CO_2_ incubator at 37°C for 12 h. The chambers were taken out, rinsed in PBS, immersed in a methanol solution at room temperature for 30 min, stained with 0.1% Crystal Violet for 20 min, and finally, the cells in the upper layer of the microporous membrane were removed carefully using cotton buds. The Transwell chambers were photographed and observed under an inverted optical microscope. Four fields were selected randomly, and the number of transmembrane cells and the mean value were counted. The experiment was repeated three times.

### Flow cytometry

Forty-eight hours after transfection, the cells were collected, digested by 0.25% trypsin, and the cell density was adjusted to 1 × 10^6^ cells/ml. Cells (1 ml) were selected and centrifuged at a rate of 1500 rev/min for 10 min, and the supernatant was discarded. Two milliliters of PBS was added to per milliliter of cell suspension, followed by centrifugation and discarding supernatant. Next, the cells were fixed after adding precooling 70% ethanol overnight at 4°C. On the second day, the cells were rinsed in PBS two times. Cell suspension (100 μl) was selected and supplemented with 50 μg of propidium iodide (PI) containing RNAase, and the solution was protected from light for 30 min and filtered using a 100-mesh nylon net. Red fluorescence at 488 nm excitation wavelength was recorded by the flow cytometer (BD Biosciences, Franklin Lakes, NJ, U.S.A.) in order to detect the cell cycle.

Cell apoptosis was detected using the Annexin V-FITC/PI double staining. The treated cells were placed in a 5% CO_2_ incubator at 37°C for 48 h, and then cells were collected and rinsed two times in PBS, centrifuged and resuspended in 200 μl of binding buffer. Cells were supplemented with 10 μl of Annexin V-FITC (ab14085, Abcam, Inc, U.S.A.) and 5 μl of PI. Three hundred microliters of binding buffer was added to the solution after gentle mixing in the dark at room temperature for 15 min. Flow cytometry (BD Bioscience, FL, NJ, U.S.A.) was used in order to record cell apoptosis at 488 nm excitation wavelength.

### Statistical analyses

Statistical analyses were performed using the SPSS 21.0 software (SPSS, Chicago, IL, U.S.A.). Measurement data were presented as mean ± standard deviation. Data differences between two groups were analyzed by *t*-test, and comparisons among multiple groups were analyzed by one-way analysis of variance (ANOVA). *P*<0.05 was considered to be statistically significant.

## Results

### Pathological observation of cells of normal skin and SCC skin tissues

The result showed that epidermic cells in the normal group were reconstituted compactly and in a uniform manner. The SCC skin cells in the SCC group showed hyperkeratosis, accompanied by parakeratosis and protuberances in the parts connecting the cutaneous horns. A significant number of SCC nests were observed in the superficial dermis, which could be seen in the horn cyst and horn pearl. In addition, heteromorphism of cancer cells was apparent (Figure 1).

**Figure 1:** Pathological observation results of skin cells in the normal and SCC groups (amplification ×200)

### The expression of Gadd45a protein in normal skin and SCC skin tissues

The percentage of positive cells of Gadd45a protein showed brown granules in the nucleus and cytoplasm (Figure 2A). The percentage of positive cells of Gadd45a protein in the normal group was 10.58 ± 1.58%, significantly lower than the SCC group (43.33 ± 3.55%) (*P*<0.05) (Figure 2B).

**Figure 2:** Percentage of positive cells of Gadd45a protein in the normal and SCC groups (**A**) Results of immunohistochemistry; (**B**) percentage of positive cells of Gadd45a protein in the normal and SCC groups; *, compared with the normal group, *P*<0.05.

### The levels of miR-374, Gadd45a, P53, P73, P16, c-myc, Bcl-2, Bax, caspase-3, and caspase-9 in normal skin and SCC skin tissues

qRT-PCR and Western blotting were employed in order to detect the levels of Gadd45a, P53, P73, P16, c-myc, Bcl-2, Bax, caspase-3, and caspase-9 and the level of miR-374 in normal skin and SCC skin tissues (Figure 3). The SCC skin tissues showed lower level of miR-374, P73, P16, Bax, caspase-3, and caspase-9, and higher levels of Gadd45a, P53, c-myc, and Bcl-2 compared with the normal skin tissues (all *P*<0.05). In addition, the half-life period of the wide-type P53 protein was as short as 10 min, and which was generally believed that the detectable product was MUT P53 protein.

**Figure 3:** The levels of miR-374, Gadd45a, P53, P73, P16, c-myc, Bcl-2, Bax, caspase-3, and caspase-9 in normal skin and SCC skin tissues (**A**) The levels of miR-374, Gadd45a, P53, P73, P16, c-myc, Bcl-2, and Bax determined using qRT-PCR. (**B**) The gray values of Gadd45a, P53, P73, P16, c-myc, Bcl-2, Bax, caspase-3, and caspase-9 protein bands, evaluated using Western blot assay. (**C**) The protein levels of Gadd45a, P53, P73, P16, c-myc, Bcl-2, Bax, caspase-3, and caspase-9 measured using Western blot assay; *, compared with the normal skin tissues, *P*<0.05; miR-374, microRNA-374.

### Gadd45a is a target of miR-374

Biological prediction website, www.microRNA.org, predicted that miR-374 can regulate Gadd45a gene at target, in addition to identifying Gadd45a as a target gene of miR-374. Results of the dual-luciferase reporter gene assay showed that luciferase activity of Wt-miR-374/Gadd45a co-transfection in the miR-374 mimics group was significantly decreased (*P*<0.05); while luciferase activity of Mut-miR-374/Gadd45a co-transfection in the miR-374 mimics group had no significant difference compared with the NC group (*P*>0.05), which indicates that miR-374 can specially bind to Gadd45a (Figure 4).

**Figure 4:** Confirmation of Gadd45a as a target of miR-374 by the dual-luciferase gene reporter (**A**) Predicted RNA-binding sites of miR-374 in Gadd45a 3′-UTR; (**B**) detection of luciferase activity; *, compared with the NC group, *P*<0.05; NC, negative control.

### *In vitro* levels of miR-374, Gadd45a, P53, P73, P16, c-myc, Bcl-2, Bax, caspase-3, and caspase-9 in each cell group

The results of qRT-PCR and Western blot assay (Figure 5) show that A431 cell line and SCL-1 cells follow similar trends. Furthermore, A431 and SCL-1 cells showed decreased levels of miR-374, P73, P16, Bax, caspase-3, and caspase-9, and increased levels of Gadd45a, P53, c-myc, and Bcl-2 compared with normal skin cells (all *P*<0.05). Compared with the blank and NC groups, the miR-374 inhibitors group had decreased levels of miR-374, P73, P16, Bax, caspase-3, and caspase-9, and increased levels of Gadd45a, P53, c-myc, and Bcl-2. The miR-374 mimics group exhibited elevated levels of miR-374, P73, P16, Bax, caspase-3, and caspase-9, and reduced levels of Gadd45a, P53, c-myc, and Bcl-2. The miR-374 inhibitors + siRNA–Gadd45a group also showed decreased level of miR-374. The siRNA–Gadd45a group presented enhanced levels of P73, P16, Bax, caspase-3, and caspase-9, and dropped levels of Gadd45a, P53, c-myc, and Bcl-2.

**Figure 5:** The levels of miR-374, Gadd45a, P53, P73, P16, c-myc, Bcl-2, Bax, caspase-3, and caspase-9 in normal cells, and A431 and SCL-1 cells in blank, NC, miR-374 mimics, miR374 inhibitors, siRNA–Gadd45a, and miR-374 inhibitors + siRNA–Gadd45a groups (**A**) The levels of miR-374, Gadd45a, P53, P73, P16, c-myc, Bcl-2, and Bax in A431 cells, measured by qRT-PCR. (**B**) The levels of miR-374, Gadd45a, P53, P73, P16, c-myc, Bcl-2, and Bax in SCL-1 cells, measured using qRT-PCR. (**C**) The gray values of Gadd45a, P53, P73, P16, c-myc, Bcl-2, Bax, caspase-3, and caspase-9 protein bands for A431 cells, evaluated using Western blot assay. (**D**) The gray values of Gadd45a, P53, P73, P16, c-myc, Bcl-2, Bax, caspase-3, and caspase-9 protein bands for SCL-1 cells, evaluated using Western blot assay. (**E**) The protein levels of Gadd45a, P53, P73, P16, c-myc, Bcl-2, Bax, caspase-3, and caspase-9 in A431 cells, determined using Western blot assay. (**F**) The protein levels of Gadd45a, P53, P73, P16, c-myc, Bcl-2, Bax, caspase-3, and caspase-9 in SCL-1 cells, determined using Western blot assay; *, compared with the normal cells, *P*<0.05; #, compared with the blank and NC groups, *P*<0.05.

### miR-374 mimics and siRNA–Gadd45a inhibited proliferation of SCC cells

The results of MTT (Figure 6) showed that A431 and SCL-1 cells follow similar trends. Compared with the normal group, cell proliferation ability in other groups was significantly improved (all *P*<0.05). There was no significant difference in cell proliferation ability among the blank, NC, and miR-374 inhibitors + siRNA–Gadd45a groups (both *P*>0.05). Compared with the blank and NC groups, the proliferation ability of SCC cells weakened in the miR-374 mimics and siRNA–Gadd45a groups with OD value dropping evidently at 48 and 72 h time periods, and the ability increased in the miR-374 inhibitors group with OD value rising evidently at 48 and 72 h time periods (all *P*<0.05). Therefore, overexpression of miR-374 and silencing of Gadd45a can inhibit proliferation of SCC cells.

**Figure 6:** Cell proliferation of normal cells, and A431 and SCL-1 cells in the blank, NC, miR-374 mimics, miR374 inhibitors, siRNA–Gadd45a, and miR-374 inhibitors + siRNA–Gadd45a groups, evaluated by the MTT assay (**A**) A431 cells; (**B**) SCL-1 cell; *, compared with normal cells, *P*<0.05; #, compared with the blank and NC groups, *P*<0.05.

### miR-374 mimics and siRNA–Gadd45a inhibited migration of SCC cells

The abilities of cell migration in each group after transfection were shown in Figure 7, and the results show that A431 and SCL-1 cells follow similar trends. Compared with the normal group, cell migration ability significantly improved and the cell healing rate decreased in the other groups (all *P*<0.05). There was no significant difference in cell migration ability among the blank, NC, and miR-374 inhibitors + siRNA–Gadd45a groups, as well as between the miR-374 mimics and siRNA–Gadd45a groups (all *P*>0.05). The miR-374 mimics and siRNA–Gadd45a groups showed weakened migration ability and increased cell healing rate compared with the blank and NC groups, while the miR-374 inhibitors group showed opposite trends (all *P*<0.05). Therefore, overexpression of miR-374 and silencing of Gadd45a can inhibit migration of SCC cells and increase the *in vitro* cell healing rate.

**Figure 7:** Cell migration of normal cells, and A431 and SCL-1 cells in the blank, NC, miR-374 mimics, miR374 inhibitors, siRNA–Gadd45a, and miR-374 inhibitors + siRNA–Gadd45a groups, evaluated by the scratch test (**A**) A431 cell migration images; (**B**) SCL-1 cell migration images; (**C**) healing rate for A431 cells under the microscope (×100); (**D**) healing rate for SCL-1 cells under the microscope (×100); *, compared with normal cells, *P*<0.05; #, compared with the blank and NC groups, *P*<0.05.

### miR-374 mimics and siRNA–Gadd45a inhibited invasion of SCC cells

The abilities of cell invasion in each group after transfection were shown in Figure 8, and the results show that A431 and SCL-1 cells follow similar trends. Compared with the normal group, the number of cells transferred from the apical chamber to the basolateral chamber was increased in other groups (all *P*<0.05). There was no significant difference among the blank, NC, and miR-374 inhibitors + siRNA–Gadd45a groups in the number of cells that transferred from the apical chamber to the basolateral chamber, as well as between the miR-374 mimics and siRNA–Gadd45a group (all *P*>0.05). Compared with the blank and NC groups, the number of cells that transferred from the apical chamber to the basolateral chamber was decreased in the miR-374 mimics and siRNA–Gadd45a, but increased in the miR-374 inhibitors group (all *P*<0.05). Therefore, overexpression of miR-374 and silencing of Gadd45a can inhibit invasion of SCC cells.

**Figure 8:** Cell invasion of normal cells, and A431 and SCL-1 cells in the blank, NC, miR-374 mimics, miR374 inhibitors, siRNA–Gadd45a, and miR-374 inhibitors + siRNA–Gadd45a groups, evaluated by the Transwell assay (**A**) A431 cell invasion images; (**B**) the number of A431 cells penetrating the Matrigel gel under the microscope (×200); (**C**) SCL-1 cell invasion images; (**D**) the number of SCL-1 cells penetrating the Matrigel gel under the microscope (×200); *, compared with normal cells, *P*<0.05; #, compared with the blank and NC groups, *P*<0.05.

### miR-374 mimics and siRNA–Gadd45a reduced the progression of SCC cell cycle

The cell cycle distribution in each group after transfection were shown in Figure 9, and the results show that A431 and SCL-1 cells follow similar trends. Compared with the normal group, the fraction of SCC cells in G0/G1 phase were decreased, while the proportion of SCC cells in S phase were increased in other groups (all *P*<0.05). There was no significant difference among the blank, NC, and miR-374 inhibitors + siRNA–Gadd45a groups in the cell cycle distributions (both *P*>0.05). Compared with the blank and NC groups, cells were increased in G0/G1 phase, while cells were decreased in S phase in the miR-374 mimics and siRNA–Gadd45a groups contrary to the miR-374 inhibitors group (all *P*<0.05). Therefore, overexpression of miR-374 and silencing of Gadd45a can inhibit proliferation of SCC cells.

**Figure 9:** Cell cycle progression of normal cells, and A431 and SCL-1 cells in the blank, NC, miR-374 mimics, miR374 inhibitors, siRNA–Gadd45a, and miR-374 inhibitors + siRNA–Gadd45a groups, evaluated by flow cytometry (**A**) A431 cell number and DNA content in G0/G1, S, and G2 stages; (**B**) A431 cell ratio in G0/G1, S, and G2 stages; (**C**) SCL-1 cell number and DNA content in G0/G1, S, and G2 stages; (**D**) SCL-1 cell ratio in G0/G1, S, and G2 stages; *, compared with normal cells, *P*<0.05; #, compared with the blank and NC groups, *P*<0.05.

### miR-374 mimics and siRNA–Gadd45a promoted apoptosis in SCC cells

Cell apoptosis rates in each group after transfection were shown in Figure 10, and the results show that A431 and SCL-1 cells follow similar trends. Compared with the normal group, the cell apoptosis rates significantly decreased in other groups (all *P*<0.05). There was no significant difference among the blank, NC, and miR-374 inhibitors + siRNA–Gadd45a groups in the cell apoptosis rates (both *P*>0.05). Compared with the blank and NC groups, cell apoptosis rates increased in the miR-374 mimics and siRNA–Gadd45a groups, while the rates decreased in the miR-374 inhibitors group (all *P*<0.05). Therefore, overexpression of miR-374 and silencing of Gadd45a can promote apoptosis of SCC cells.

**Figure 10:** Cells apoptosis of normal cells, and A431 and SCL-1 cells in the blank, NC, miR-374 mimics, miR374 inhibitors, siRNA–Gadd45a, and miR-374 inhibitors + siRNA–Gadd45a groups, evaluated by flow cytometry (**A**) A431 cell apoptosis, (**B**) A431 cell apoptosis rate, (**C**) SCL-1 cell apoptosis, (**D**) SCL-1 cell apoptosis rate; *, compared with normal cells, *P*<0.05; #, compared with the blank and NC groups, *P*<0.05.

## Discussion

SCC has been ranked as the sixth most common death causing cancer across the world owing to its high occurrence, lethality, and malignancy rates [14,15]. SCC is characterized by etiological, phenotypic, biological, and clinical heterogeneity [16]. Gadd45a is involved in DNA repair and replication, and cooperates with proliferating cell nuclear antigen and acts as a stress sensor regulating cellular responses to a series of stress stimulations [17,18]. The present study aims to explore the effects of miR-374 on proliferation, migration, invasion, and apoptosis of human SCC cells by targeting Gadd45a through the P53 signaling pathway. The results of a plethora of experiments show that up-regulated miR-374 can inhibit proliferation, migration, and invasion and promote apoptosis in SCC cells by down-regulating the expression of Gadd45a through the P53 signaling pathway.

As the initial discovery in the present study, the SCC group showed elevated expression of Gadd45a and P53, and decreased expression of miR-374 compared with the normal group, thus confirming elevated Gadd45a and P53 and down-regulated miR-374 can be triggered in SCC. Gadd45a plays a role in the maintenance of DNA repair and P53-dependent cell cycle checkpoints [17]. The tumor suppressor pathway P53 is essential in controlling the reaction and outcome of common cancer therapies [19]. In addition, proteins of Gadd45a and P53 are overexpressed in pancreatic cancer, which may be associated with the malignant behavior of pancreatic cancer [20]. Consistent with our study, miR-374 exhibited decreased expression in early-stage non-small cell lung cancer (NSCLC), which is associated with poor patient survival [21].

After transfection, the results of qRT-PCR and Western blot analysis revealed that miR-374 suppressed the expression of Gadd45a in order to block the P53 signaling pathway. Our study confirmed that Gadd45a was the target gene of miR-374 by dual-luciferase reporter gene assay elaborating the mechanism of miR-374 in the regulation of Gadd45a. P53 gene plays a dual role as an initiator of DNA repair and as a trigger of apoptosis, and Gadd45a gene is capable of maintaining genomic stability [20]. P53 is closely associated with DNA damage and repair by means of regulating its downstream genes such as p21 and Gadd45 [22]. In addition, P53 protein stabilization was greatly abolished following the disruption of Gadd45a [23]. The p53 signaling pathway integrates a variety of environmental stimuli and acts as the nodal point for the modulation of cell proliferation or cell death via apoptosis. In cases of head and neck SCC, patients with overexpressed p53 protein (p53+), it was found that p53 contributes to a poor outcome and poor tumor response to therapy [24]. Osman et al. [25] and their findings demonstrate that p53 phenotype is the most informative predictor of unfavorable outcomes in the larynx preservation setting in SCC of the larynx and pharynx. Moreover, P53/miR-374/AKT1 regulates the apoptosis in colorectal cancer cells as a reaction to DNA damage [26]. Zhang et al. [6] report that Gadd45a plays an important role in the metastasis of OSCC as a result of regulating the bioactivity of the tumor cell, and its distribution may be indicative of the clinical outcome of OSCC.

Our study also revealed that the miR-374 mimics and siRNA–Gadd45a groups exhibited decreased SCC cell proliferation, migration and invasion, and increased apoptosis, in contrast with the miR-374 inhibitors group, which identified that overexpression of miR-374 can inhibit cell proliferation, migration and invasion, and induce apoptosis in human SCC cell lines by down-regulating Gadd45a through the P53 signaling pathway. Mutation or loss of P53 is probably related to an increased susceptibility of cancer, and most functions of P53 have been considered to protect from malignant progression [27]. Additionally, the P53 gene is required for the proper induction of the G1 checkpoint and functions to up-regulate the growth arrest and DNA damage-inducible WAF1/p21 and Gadd45a expression. Additionally, Gadd45a, acts as a downstream mediator of P53, and is capable of deactivating P53, thereby contributing to cell cycle regulation through binding with cyclin-dependent kinases and proliferating nucleus antigen [17]. It has reported that miR-374 was decreased in glioma tissues and up-regulation of miR-374 in U87 and U251 cells inhibited the proliferation of glioma cells [28]. Furthermore, it has been demonstrated that non-thermal atmospheric pressure plasma (NTP) is capable of inducing cell apoptosis in P53 wild-type oral SCCs through a new mechanism involving DNA damage and triggering of sub-G 1 arrest via the ATM/P53 signaling pathway [29]. A previous study also suggested that miR-374 can suppress migration, proliferation, intrahepatic metastasis, and invasion in colon adenocarcinoma cell lines SW620 and HCT116 [30]. Furthermore, Huang et al. [31] report that specific miRNAs (miR-374a, miR-181a, miR-519a, and miR-630) regulated the expression of ATG16L1, ATG5, ATG10, ATG6/BECN1, and UVRAG, adding another expression level control for autophagic pathways in SCC cells.

In conclusion, our study demonstrated that miR-374 can effectively suppress Gadd45a expression in order to inhibit cell proliferation, migration, and invasion, and induce apoptosis in human SCC cell line via blocking the P53 signaling pathway. These results project miR-374 as a promising therapeutic strategy for patients suffering from SCC, and experimental verification of predicted miRNA requires further researches and analyses.

## Abbreviations

DMEM: Dulbecco’s minimum essential medium
Gadd45a: growth arrest and DNA-damage-inducible protein 45 α
GAPDH: glyceraldehyde-phosphate dehydrogenase
HE: hematoxylin–eosin
MAPK: mitogen-activated protein kinase
MTT: 3-[4,5-dimethylthiazol-2-yl]-2,5 diphenyl tetrazolium bromide
OSCC: oral squamous cell carcinoma
PBST: phosphate-buffered saline Tween-20
PI: propidium iodide
RIPA: radioimmunoprecipitation assay
SCC: squamous cell carcinoma
